# Optimization of Tree-Based Machine Learning Models to Predict the Length of Hospital Stay Using Genetic Algorithm

**DOI:** 10.1155/2023/9673395

**Published:** 2023-02-14

**Authors:** Atefeh Mansoori, Masoomeh Zeinalnezhad, Leila Nazarimanesh

**Affiliations:** ^1^Department of Industrial Engineering, Science and Research Branch, Islamic Azad University, Tehran, Iran; ^2^Department of Industrial Engineering, West Tehran Branch, Islamic Azad University, Tehran, Iran; ^3^Department of Healthcare Administration, Entrepreneur and Management Consultant, Science and Research Branch, Islamic Azad University, Tehran, Iran

## Abstract

The length of hospital stay (LOS) is a significant indicator of the quality of patient care, hospital efficiency, and operational resilience. Considering the importance of LOS in hospital resource management, this research aims to improve the accuracy of LOS prediction using hyperparameter optimization (HPO). Expert physicians and related studies were reviewed to determine the variables affecting LOS. The electronic medical records of 200 patients in the department of internal medicine of a hospital in Iran were collected randomly. As the performance of machine learning (ML) models can vary based on the characteristics of the features, several models were applied and evaluated in this study. In particular, k-nearest neighbors (KNN), multivariate regression, decision tree (DT), random forest (RF), artificial neural network (ANN), and XGBoost have been evaluated and improved. The genetic algorithm (GA) was applied to optimize the tree-based models. In addition, the dummy coding technique, sometimes called the One-Hot encoding, was used to encode categorical features to increase prediction accuracy. Compared with other algorithms, the XGBoost model optimized by GA (XGB_GA) achieved higher accuracy and better prediction performance. The mean and median of absolute errors in the test dataset for this model were 1.54 and 1.14 days, respectively. In other words, the XGB_GA model reduced the mean absolute error by 37%, which is beneficial in the reliable design of a clinical decision support system.

## 1. Introduction

Since the 1970s, the length of hospital stay (LOS) has been studied and researched to achieve better quality and performance in hospitals. Hospitals try to achieve better outcomes with the least possible resources. Developed countries evaluate the LOS as a key performance indicator to reduce healthcare costs without compromising patients' outcomes [1]. The growth in the number of patients admitted and the increase in inpatient unit costs have resulted in issues in hospital bed management. The length of stay and the lack of knowledge about the discharge time are among the complications that affect hospital bed management [2]. While the length of stay is affected by various factors that may make it difficult to predict, knowing its accurate value can significantly help manage beds and staff schedules [3]. LOS is one of the indicators of hospital quality, productivity, and performance. As a result, in dealing with issues such as planning resources, managing capacity, and staff level, LOS prediction could be an effective solution. It increases the number of patients receiving services, increases their safety, reduces healthcare costs, and helps optimize resource consumption [4]. Incorrect prediction of LOS can cause wasting and blocking bed days. It can also lead to disruption in the provision of medical services and dissatisfaction among patients and health workers.

On the other hand, accurate prediction leads to better allocation of resources and better organization of services from the time of admission to the discharge of the patient [5, 6]. LOS prediction, traditionally performed by experts, is unreliable because the patient's background information is not considered [7]. Healthcare professionals assign different LOS to a patient; therefore, the assigned LOS depends on the predictor, not the patient. Hence, the automatic prediction of LOS is valuable and significant [8]. Apart from the future planning for the use of beds, LOS estimation is also helpful for the scheduling of specialists and human resources, determining the appropriate insurance plan and reimbursement system in the private sector, and preparing the patient's relatives to plan for the return of their patients [9].

A recent review revealed that worldwide scientific attempts for accurate LOS prediction over the past fifty years have led to a rise in the number of related publications, suggesting the importance of this topic. Many publications provide a model for LOS and focus on the best statistical technique to provide the most accurate results. The latest studies, however, move toward more sophisticated methods, such as machine learning (ML), rather than regression [8]. The focus of the literature has been chiefly on proposing innovative prediction methods. Alahmar et al. proposed a stacked-ensemble method combining the result of different models to improve performance [10]. In a similar study, Muhlestein et al. came up with another ensemble approach for ranking the result of different models to select the most accurate one [11]. Danilov et al. have applied a deep learning algorithm, the RNN-GRU, for text-mining operative reports [12]. Although the regression technique is still used for prediction purposes [13–15], many studies applied various ML techniques to compare their result and find the most accurate one for their prediction purpose [4, 16, 17].

Related works can also be classified in terms of the type of studied sample. Various types of hospital units, such as intensive care units (ICUs) [14, 18] and newborns units [4, 19], as well as different medical diagnoses, were studied, including COVID-19 patients [20] and lung cancer [21]. Although the methods used in the literature have yielded good results, the hyperparameter tuning problem still exists in the modeling procedure [4, 16, 18, 20, 21]. There are two types of parameters in ML models, those learned during the training process and hyperparameters, such as maximum depth in a decision tree. Finding the optimal setting of hyperparameters is called hyperparameter optimization (HPO) [22]. Some algorithms have many hyperparameters making the HPO more complicated. Studies have shown the impact of HPO on performance improvement. By HPO, we mean that we are looking for optimal performance using the tuned hyperparameters of the model. The least complicated method is manual tuning. Manual search is a demanding task in terms of time and effort, and since there are many possible settings, this solution needs to scale. Some well-known alternative methods are grid search and random search, performing Bayesian optimization and heuristic approaches such as GA [23].

Another issue worth noting in the literature is the occasional use of the XGBoost algorithm. When applied to structured data, XGBoost is popular and capable of powerfully solving large-scale ML problems, and it outstands many other complex ML algorithms. Its high accuracy and many hyperparameters can be mentioned to outline good reasons for choosing XGBoost over other alternatives [23]. It is suitable for large-scale datasets due to its parallel integration mechanism and has regularization promotion characteristics. It is also highly accurate and interpretable [24]. A well-tuned XGBoost can provide better prediction results than a poorly configured XGBoost. Therefore, it is beneficial to improve XGBoost in a time-efficient way rather than doing the calculation manually [23]. The XGBoost model, which has many applications in the field of data science and has achieved many successes in other areas, has rarely been used in LOS prediction. Chen has proposed a “nonlinear weighted XGBoost” model to predict LOS as a classification problem and grid search for HPO. The model presented by Chen has the highest accuracy compared to other models, such as the support vector machine (SVM) [24]. Budholiya et al. utilized an optimized XGBoost classifier to predict heart disease. To optimize the hyperparameters of XGBoost, they used Bayesian optimization and achieved a prediction accuracy of 91.8% [25]. Other examples of XGBoost applications in other areas include early detection of sepsis in ICU [26], early diagnosis of heart disease [27], diagnosis of chronic kidney disease [28], prediction of the groundwater level [29], and breast cancer prediction [30].

The XGBoost model has 25 hyperparameters, each of which has its function and makes the optimization process an extremely complicated problem [31]. Proper hyperparameter tuning is essential for the successful application of any predictor [25]. The HPO process is computationally challenging. It involves multiple training cycles of the ML model, and the dimension of the problem increases with the increase in the number of hyperparameters. Bayesian optimization is explicitly designed to minimize the number of necessary training cycles in the grid search method; however, it cannot deal with high-dimensional searches when many hyperparameters are involved. Larger datasets add to the training time and the complication of the problem too. A user-defined search space for hyperparameters is required for many tuning approaches, which is impossible in practical cases due to the user's lack of knowledge. As such, a primary barrier to the broader use of HPO techniques is setting the search bounds of hyperparameters [22].

Although other studies have achieved good results in LOS prediction by using a wide range of ML methods, only some have explored XGBoost or HPO. The primary issues in hyperparameter tuning of ML models are time efficiency and space search. Bayesian optimization improves the time efficiency of the grid search method, yet it works with a limited search space such as the grid search method. On the other hand, GA has overcome both issues, i.e., it searches over a broader range of spaces in a more time-efficient manner. Due to its high robustness, the GA helps the XGBoost model to become more stable and fit better [31]. It is also a more efficient solution to the search space-defining problem and the computational cost of HPO. Using the GA helps to rapidly evaluate a broader range of solutions in order to find the best options. This issue is crucial for designing a clinical decision support system and big data analysis.

The use of GA to optimize XGBoost hyperparameters is seen in studies with different scopes. Jiang et al. used this technique to detect pedestrians [32], and Feng et al. used it to predict terrorist attacks [31]. However, this technique is yet to be used to improve the XGBoost model in the field of LOS prediction. This study proposes integrating the GA and XGBoost (XGB_GA) to predict LOS with higher accuracy. The proposed algorithm considers the HPO as an optimization problem; i.e., the algorithm is looking for the optimum value of the hyperparameters so that the mean square error (MSE) function of XGBoost is minimized. As a result, the accuracy of the prediction improves while the computational cost is reduced.

It is clear from the reviewed studies that addressing regularization and underfitting/overfitting problems is needed [25]. Limited previous techniques provided considerable improvement in the results; however, there still exist some techniques which remain unexplored, particularly in the LOS prediction: (i) previous approaches have rarely explored tree-based ML algorithms such as XGBoost, which have several parameters for handling underfitting/overfitting and regularization; (ii) the general approaches have not used categorical feature encoding methods to encode categorical features in the LOS dataset; (iii) the previous methods have not used GA as an HPO technique for optimizing ML models for better prediction of LOS; (iv) the previous studies have rarely researched a hospital's department of internal medicine to develop its own LOS predictive model; and (v) limited research has predicted the absolute value of LOS and they have only used one model. Hence, this research uses k-nearest neighbors (KNN), multivariate regression, tree-based ML algorithms, artificial neural networks (ANNs), and genetic algorithm (GA) to design an accurate model to predict the absolute value of LOS. The significant contribution of the study includes the following:

- Exploring the application of tree-based ML algorithms, including XGBoost, in the LOS prediction
- Using the one-hot encoding method to encode categorical features in the LOS dataset
- Applying GA for hyperparameter optimization of XGBoost, decision tree, and random forest to increase the accuracy of prediction
- Investigating the hospital's department of internal medicine to develop its own LOS predictive model
- Predicting the absolute value of LOS using several data mining algorithms

The organization of this study is as follows. In Section 2, LOS prediction literature and standard HPO techniques are discussed. In Section 3, data collection, data preprocessing, model training, and HPO are presented.  Section 4 describes the results, and the conclusion is presented in Section 5.

## 2. Related Works

In this section, LOS prediction in the literature is discussed. First, studies have been evaluated from different points of view, including the studied sample, prediction method, results, and approaches used for hyperparameter tuning. The second section discusses standard HPO methods and their advantages and disadvantages.

### 2.1. LOS Prediction

The three primary categories of LOS prediction methods are (1) regression model, (2) ML, and (3) deep learning, which is a subcategory of ML [8]. For example, Baek et al. fitted a multivariate regression model on all hospital inpatient information, and the *R*^2^ value for their model was 0.267 [13]. Like Beak et al., Ray-Zack et al. predicted the LOS of radical cystectomy for muscle-invasive bladder cancer patients with a multivariate regression model. The *R*^2^ value reported for the regression model was 0.048 [15]. Meadows et al. built a logistic regression model to predict short-term (less than 48 hours) and long-term (more than 48 hours) hospitalization of ICU patients following cardiac surgery with an accuracy of 79% [14].

Alahmar et al. applied the stacked-ensemble method to predict the LOS of diabetic patients [10]. Their new proposed method showed the best performance (accuracy 0.81) compared to nonensemble models, including regression-based, tree-based, and ANN models. However, the results showed that the improvement achieved by the ensemble method compared to the random forest model (accuracy 0.80) and the gradient boosting method (accuracy 0.80) was insignificant. To optimize the selected hyperparameters, they performed the manual HPO.

Thompson et al. explored a newborns unit dataset to predict LOS using methods such as Naïve Bayes, logistic classifier, multilayer perceptron, SVM, decision tree (J48), and random forest [17]. They used 10-foldcross-validation and achieved the highest accuracy of 0.87 using random forest but did not mention the hyperparameter tuning process. Daghistani et al. applied random forest, SVM, Bayesian network, and ANN to predict the LOS of cardiac patients and reported the highest accuracy of 80% from random forest [4]. The hyperparameter tuning issue could also be noticed in this research study.

Using an innovative solution, Danilove et al. applied deep learning algorithms, the RNN-GRU, for text-mining operative reports of neurosurgery patients to predict their LOS as a continuous variable. The mean absolute error (MAE) resulting from the proposed method was 2.8 days [12]. Muhlestein et al. used brain surgery data and developed a new approach that systematically ranks different ML models [11]. The new technique selects the best models automatically and achieves the optimal answer by combining the results. The strength of this research is the increase of RMSLE in predicting the test dataset (0.63) compared to the training dataset (0.55) although model hyperparameters were optimized using the grid search method.

Steele and Thompson have addressed LOS prediction for better planning of the hospitalization of elective patients. They constructed the prediction model using Naïve Bayes, Bayesian network, KNN, kstar, locally weighted learning, C4.5 decision tree, SVM, and decision table. The Bayesian network has the best accuracy (0.9) among other models, and their research did not discuss hyperparameter tuning [16]. In another study, Abd-Elrazek et al. used ML models such as fuzzy logic, KNN, Naïve Bayes, random forest, SVM, and ANN to predict the LOS of ICU patients. Fuzzy logic had the best prediction results, followed by random forest, with an accuracy value of 0.92 and 0.9, respectively. Parameter tuning was not mentioned in the modeling process [18]. Mahboub et al. used the decision tree model to predict the LOS of COVID-19 patients. The MAE reported for this model was 2.8 days, and no other method was applied to compare the results with [20].

In a study, Chen investigated the performance of the nonlinear weighted XGBoost model compared to other ML models in predicting LOS. To optimize the hyperparameters of the XGBoost, the K-CV method was used with a value of *K* = 3. In all the models considered in this work, only four values were investigated for each hyperparameter. The results showed that the nonlinear weighted XGBoost model was the most accurate among all models, and its RMSE value was 1.52 days [24]. Similarly, Alsinglawi et al. developed logistic regression, random forest, and XGBoost models to predict the LOS of lung cancer patients hospitalized in the ICU. The random forest has shown the best performance among other models. Hyperparameter tuning and evaluating the models have not been performed in this study. Consequently, the reported results were based on the training dataset [21].

Table 1 shows a summary of the studied literature chronologically. The table gives a better view of different aspects of LOS perdition in similar studies. In terms of the studied sample, it can be observed that previous studies rarely researched a hospital's department of internal medicine to develop LOS predictive models. Limited research predicted the absolute value of LOS and those that developed models for LOS's absolute value prediction using only one method. Previous approaches have hardly explored tree-based ML algorithms such as XGBoost, which have several parameters for handling underfitting/overfitting and regularization. In addition, there needs to be a report on using GA as an HPO technique for optimizing ML models for faster prediction of LOS.

### 2.2. Hyperparameter Optimization Methods

Grid search is a prevalent method in which the user manually defines a subset of hyperparameters for a target ML algorithm, and the method searches through that subset. Despite straightforward implementation and parallelism capabilities that make grid search a reliable method in low-dimensional spaces (i.e., 1D or 2D), the computational cost increases dramatically as the number of hyperparameters increases [23].

In random search, a generative process defines the configuration space and draws random samples, and this random sample assigns the hyperparameter and evaluates them. Random search and grid search have common advantages; however, random search is more efficient in high-dimensional spaces, and generally, random search performance is better than grid search [23].

For objective functions that are slow and costly to evaluate, Bayesian optimization is a powerful strategy that tries to predict the performance of untested combinations [23, 33]. Compared to grid search, Bayesian optimization is more dynamic and requires two key components to function. Those components are the probabilistic surrogate model and the acquisition function. The role of the surrogate model is to be fitted to all the target function observations made so far. Then, the acquisition function looks for parameters that improve the search process to find the most optimum hyperparameters.

The GA is one of the population-based metaheuristic optimization algorithms developed with inspiration from the theory of natural selection. In this algorithm, a new population is generated by repeatedly using genetic operators on each individual in the population. The critical elements of this algorithm are chromosomes, selection, crossover, mutation, and fitness function. The general performance of this algorithm is as follows: Initially, the population *Y* (*Y* is the number of answers or solutions) consisting of *n* chromosomes (*n* is the number of parameters of the problem) is randomly generated. Two chromosomes (two answers or two solutions), namely, C1 and C2, are selected from the population based on their fitness. C1 and C2 will produce the new offspring O with the crossover operator. The probability of this operation would be CP, which is the crossover probability parameter. The genetic mutation operator with the probability of MP is then applied to *O* to generate a new member *O*'. Member *O*' is added to the previous population to form a new population. The selection, crossover, and mutation process continue until an entire population is generated. The probability of crossover and mutation is why the GA can dynamically search for the optimal solution and reach it [34].

## 3. Materials and Methods

### 3.1. Data Source

The studied hospital in this research has 300 beds and 1055 physicians and staff. The hospital provides clinical and paraclinical services and has 19 inpatient departments. It has a health information system to collect and store patients' data. The information studied in this research was extracted from the department of internal medicine.

In order to determine the variables that may affect LOS and collect the necessary data, similar studies were reviewed. Two hundred records of electronic data of 100 men and 100 women were randomly extracted from the information system.  Table 2 shows the variables used in this study, including age, sex, type of insurance, marital status, medical advice number, and physician's expertise level.

### 3.2. Data Preprocessing

The data were checked, and there were no missing values. The mean age of the patients was 63 years, with a standard deviation of 19 years. 50% of the data were related to women, and 50% were related to men. 90% of patients were married, and others were single. The average number of medical advice numbers was two, with a standard deviation of 3. The LOS had a mean value of 5.6 days and a standard deviation of 3.4 days. The primary insurance type and physician's expertise level variables had relatively unbalanced distributions. 90% of the patients had ordinary social security insurance, and the rest were in other insurance groups. 45% of the patients were treated by general practitioners, 54% by specialists, and the remaining 2% by subspecialists.  Table 3 shows the statistical characteristics of each variable.

Dummy coding, sometimes called “one-hot encoding,” was used to turn the categorical variables into numerical variables. In order to remove outliers, data with 1.5 times IQR (interquartile range) greater and less than the first and third quartiles were removed from the data. The lower limit value of outliers was calculated as −0.5, and the upper limit value was 11.5. Therefore, patients with LOS of more than 11.5 days (eight records of data) were excluded from the data.

Since ML algorithms cannot analyze categorical data, the one-hot encoding technique creates binary variables representing the old categorical variable. The ML algorithm can then process these new binary variables [35]. In one-hot encoding, a new feature is created for each category level, and a binary feature is created [25]. One-hot encoding of four categorical variables is shown in Figure 1. For each category of a categorical variable, one variable (one dimension) is added to the variables, and the value of this new variable in each row is set to 0 or 1. The value of the dummy variable is 1 when the original categorical variable is the same as the created dummy variable, and it is zero for other cases. Finally, the original categorical variable and its records are removed from the data.

Pearson correlation analysis has been performed, and the coefficients are reported in Table 4. According to Table 4, LOS has the highest positive correlation, with a *p* value of less than 0.05, with the medical advice number of 0.46, primary insurance type_employee health insurance of 0.2, and physician expertise level_subspecialty physician of 0.17. The highest negative correlation, with a *p* value of less than 0.05, is with the primary insurance type_without insurance variable (−0.16). Other correlation values were insignificant, and their *p* valuewas greater than 0.05; nevertheless, they were not removed from the dataset to check their impact on the output of the models. The dataset was divided into training and test sets in the last step. 85% of the data was assigned to the training dataset and 15% to the test dataset. The data distribution was checked in each dataset, and both had relatively the same distribution. This control mattered since the data were unbalanced.

### 3.3. Model Training

The models used in this work include KNN [18], multivariate regression [36], decision tree [37], random forest [4], ANN [38], and XGBoost [39] so that the results of the improved model can be compared. All models were built in Python version 3.8.5. The number of parameters in the KNN model (the number of neighbors) was estimated at 12. The estimation was performed with the help of the K-CV method with a value of *k* = 10. The regression model was built in two forms. First, one was built with all variables on LOS. After checking the regression assumptions, the natural logarithm of LOS was calculated and added to the data. Another multivariate regression model was built on transformed LOS, which hereafter will be known as a transformed regression model. Regression and transformed regression models were rebuilt based on *t*-test results with a *p* value of less than 0.05 and evaluated on the test dataset. These two models will be referenced with the names Lm and Lm_transformed, respectively. Since changing LOS to the natural logarithm of LOS improved the regression assumptions and brought the data closer to the normal distribution, other models were also built using the natural logarithm of LOS. Decision tree (DT_default), random forest (RF_default), and XGBoost (XGB_default) were built on the training dataset using default hyperparameter values. The ANN model was built with a 2-layer structure. Twelve neurons were placed in the first layer and six in the second layer. Finally, the evaluation of the models was performed on the test dataset. The details of default hyperparameters of tree-based models are presented in Table 5.

### 3.4. Optimization with the Genetic Algorithm

The values set for the hyperparameters of the tree-based models are based on the default values in the libraries developed for Python (see Table 5). Different combinations of the mentioned hyperparameters can be used in the models. In this research study, the PyGAD module and the PyGAD.GA class developed for Python were used to apply the GA for HPO [40].

Implementing the GA for each model has three basic steps: determining the fitness function, determining the range of hyperparameters of each model to be evaluated in the GA, and specifying the parameters of the GA. The fitness function for each model is the mean squared error (MSE) calculated with the K-CV method and *k* = 5 to reduce the overfitting of the model on the training data [31].

The hyperparameter space of each model that needs to be checked by the GA is as follows. For the decision tree model, the maximum depth of the tree is set between 1 and 1000. The higher value of max_depth leads to more tree expansion and overfitting on the data. The minimum number of samples per node is between 1 and 50. The alpha value is between 0 and 1. When ccp_alpha equals zero, no pruning occurs, and higher values lead to more pruned trees.

For the random forest model, the maximum tree depth is between 1 and 7, and the minimum number of samples per node is between 1 and 50. These two hyperparameters have the same function as in the decision tree. The number of variables that should be used in constructing each tree is between 1 and 12. It ranges from one to the maximum number of features which in our problem is 12. The number of trees is considered to be between 50 and 1000, as fewer trees will provide inaccurate results.

On the other hand, too many trees will add to the training time while no improvement happens. The maximum number of samples, defined as the number of samples to draw from *X* to train each base estimator, is set between 0.1 and 1. We are looking for its optimum value that ranges from 10% to 100%.

In the XGBoost model, the learning rate is between 0.001 and 1. The learning rate is the step size shrinkage used in the update to prevent overfitting. The number of trees is set between 50 and 1000. The maximum depth of the tree is between 1 and 7. The percentage of samples (subsample) and variables (colsample_by_tree) used in constructing each tree is between 0.1 and 1. The subsample is the ratio of the training instances, and it will prevent overfitting. Subsampling will occur once in every boosting iteration. Setting it to, for example, 0.1 means that XGBoost would randomly sample 10% of the training data before growing trees. Colsample_by_tree is the subsample ratio of columns when constructing each tree. Subsampling occurs once for every tree constructed. The regularization term is considered between 1 and 3. Increasing this value will make the model more conservative [31]. The hyperparameter space of each model that the GA should check is also presented in Table 5. The evaluation result of the decision tree, random forest, and XGBoost model that improved by utilizing the GA will be referenced with the names DT_GA, RF_GA, and XGB_GA, respectively.

GA parameters include the number of generations or the ending condition of the algorithm, the number of parents that the crossover operator must use, the number of solutions or individuals in each population, the type of selection operator, the type and probability of the crossover operator, and the type and probability of mutation operator. GA parameters must be determined before running the algorithm. For this purpose, the number of generations is 50, the number of parents who can participate in the crossover operation is 2, and the number of solutions (individuals) in the population is 20. The type of selection operator is steady state, the type of crossover operator is uniform with a probability of 60%, and the type of mutation is random with a probability of 1% [31]. Implementing the GA algorithm to optimize the hyperparameters of a tree-based model is shown in Table 6.

## 4. Results and Discussion

### 4.1. Prediction Accuracy Analysis

The models detailed in the previous section were evaluated on the test dataset, and absolute errors were calculated for each model. The statistical indices of absolute errors, including mean, median, standard deviation (SD), interquartile range (IQR), minimum (min), and maximum (max), are reported in Table 7.

The lowest mean absolute error (MAE) is 1.52 days and belongs to the transformed regression (Lm_transformed). With a slight difference from that, the improved XGBoost (XGB_GA) model has the lowest MAE value, equal to 1.54 days. After that, the lowest MAE belongs to the regression model called Lm (1.56 days), ANN (1.61 days), RF_default (1.65 days), RF_GA (1.76 days), KNN (1.78 days), DT_GA (1.95 days), DT_default (2.15 days), and finally the XGBoost_default (2.45 days).

A lower MAE generally means better model accuracy, but MAE alone does not answer the question of which model is the best. In order to solve this problem, it is better to check the error dispersion indices. These indices include the median, SD, and the IQR of the absolute errors in addition to the MAE. Dispersion indices help to have a better view of the model performance on each data record in the test dataset. The lowest median belongs to the RF_default (1.02 days), followed by the XGB_GA (1.14 days). The lowest standard deviation belongs to Lm and ANN, with values of 1.14 and 1.20, respectively. The smallest IQR belongs to a DT_default (1 day) and XGB_GA (1.26 days). Since there are three dispersion indices for ranking the models, the average of all these three indices was calculated for each model in order to determine which model has the most negligible dispersion error in the test dataset. This ranking puts the XGB_GA model in the first place and the Lm_transformed in second place. After that, Lm, ANN, RF_GA, RF_default, DT_default, KNN, DT_GA, and XGB_default, respectively, have the lowest value in dispersion indices. This ranking means that we are not only looking for a model with lower prediction errors on average but also we look for more records of data that are predicted as accurately as possible. In other words, if we draw the range of errors of each model in a boxplot diagram, we want to see more compression in its diagram.

Figure 2 depicts the given explanations about the error comparison of the models in a boxplot diagram. As shown in the figure, the XGB_GA boxplot has the most compression among the rest of the models. After that, the Lm_transformed model has this position. The MAE of these two models is the lowest among the others. Another indicator that should be assessed in the analysis of each model is the maximum prediction error. In this case, the Lm_transformed model and the ANN have the lowest value. However, the graphs in Figure 2 show that in highly accurate models such as XGB_GA and Lm_transformed, the number of cases predicted with a high error is small. For example, for the XGB_GA, this term is 2 out of 29 cases, which is about 6% of the data.

In addition to comparing models and checking their prediction accuracy, it is necessary to address the effect of GA performance. Table 7 shows that the GA has reduced all the error indicators in the XGBoost model by at least 25%. In decision tree and random forest, the changes have been slightly different. In the decision tree, all error indicators have improved except IQR, which increased by 100%. The mean, median, standard deviation, and maximum error have been reduced to 10%, 17%, 10%, and 9%, respectively. In the random forest, the mean and median errors increased by 7% and 31%, respectively. The standard deviation, IQR, and maximum error decreased by 4%, 20%, and 2%, respectively. In other words, the boxplot of errors in Figure 2 is more compressed (see Table 8).

Another tool that helps to compare the performance of the models and the GA effect is the graph of predicted values (*Y*-axis) versus actual values (*X*-axis). Ideally, the data in this graph should fit on a 45-degree line, meaning that the predicted value is precisely the same as the actual value; however, it is impossible in practice. Models whose values have less dispersion around the diagonal line are considered better ones. The reason behind the lower MAE and error dispersion in the XGB_GA and Lm_transformed can be seen in Figure 3. Although it is difficult to compare the models in this type of diagram, the way the tree-based models change after using the GA can be seen. The MAE value of the decision tree model decreases while the error dispersion values for the random forest model increase. The improvement in the XGBoost model is notable as the values approach the diagonal line.

### 4.2. Discussion

In conclusion, if the order of accuracy of the models is considered (see Figure 4), the Lm_transformed and XGB_GA models have an excellent ability to predict LOS. After those two models, Lm, ANN, RFs, KNN, DTs, and XGB_default have the best prediction accuracy, respectively. The XGB_default and both DT models are among the weakest models. Their result is even weaker than the base model, KNN. A weaker result was expected from the DT models than others employing ensemble learning. Figure 4 shows the error values of the models, which are arranged relatively for comparison in the order of the MAE. The diagram in Figure 4 helps to compare the models and check the trend of the error indicators. The graph shows that the models become weaker in the mentioned order, thereby decreasing their accuracy. In other words, the error values increase in them.

The noteworthy point about the first two models is the competition between the complex tree-based model optimized with metaheuristic methods (XGB_GA) and the simple transformed regression model (Lm_ transformed). The XGB_GA model has a higher mean but lower error dispersion than the Lm_transformed model. Since the difference in the MAE of these two models is insignificant, the XGB_GA model can be chosen as the most accurate one.

There are two important points regarding the two top models in this research. One is their interpretability and the other is their computational process. The regression model has better interpretability than the XGB_GA model because it is possible to check which variable, and to what extent, will affect the output. At the same time, this possibility is not available for the XGB_GA model. The regression model was based on *t*-test results and variables selected by the user's decision. The XGB_GA model is immune from the user's intervention in creating the model, and no variable or data is removed during the process.

To conclude, XGB_GA has three critical advantages over other models. The first is the lowest value of MAE, the second is the lowest value of prediction error dispersion, and the third is the absence of analyst involvement in decision-making and creating the final output. The median value of XGB_GA is 1.14 days, and the third quartile of the error is less than two days, meaning that the model predicts LOS with less than two days of error in 75 percent of cases. For a future decision support system, a model that is less dependent on the intervention of the researcher or analyst can be a better choice. In most cases, the model must also predict LOS with a minor error. Therefore, XGB_GA could be selected as the best model.

As a criterion for measuring the accuracy of the models, we can rely on the reported results of other researchers. For this purpose, those studies that predicted the absolute value of LOS and reported RMSE or MAE indices can be included for comparison. Danilov et al. reported the MAE for their proposed model to be 2.8 days. They applied text-mining techniques to operative reports with deep learning methods [12]. Mahboub et al. also reported a value of 2.8 days as the MAE of the decision tree model for predicting the LOS of COVID-19 patients. Chen reported an RMSE value of 1.52 days for the nonlinear weighted XGBoost model, whose hyperparameters were optimized using a grid search method. Therefore, the models presented in this research study have had acceptable results compared to the existing literature. At least, this has been the case with MAEs. The best model in this research had an MAE of 1.54 days and the worst model had an MAE of 2.45 days. However, since the error dispersion indices were not reported in similar research, it is impossible to compare and judge the results from this perspective.

The main issue this research tried to study was the effect of GA in improving ML model results. The GA was used to calculate the optimal hyperparameters of the decision tree, random forest, and XGBoost models. The positive effect of the GA on the XGBoost model is undeniable. It has reduced all the error indicators. Considering the value of the error indicators, the error distribution, and the related graphs, the decision tree model has become weaker, and the random forest model has generally improved. The random forest model has generally improved. Graph (e) in Figure 3 shows that the optimized decision tree only fitted a constant number on the data to reduce the MAE. A constant value as the final model is considered a poor result since every case will have the exact prediction regardless of the input variables. In Figure 3(j), for the RF_GA model, the general form of data dispersion is similar to Figure 3(i)—RF_default. The only difference is that the data are closer to the diagonal line, which means that the random forest model has improved after optimization.

## 5. Conclusions

This study aimed to improve the LOS prediction accuracy by focusing on the HPO process. Literature shows that this procedure has been neglected in most similar studies. Due to its superiority over other standard methods, GA has been selected for this purpose. In this work, the impact of GA on performance improvement was tested experimentally by integrating it with one of the most accurate ML models, XGBoost. The newly proposed method outperformed other modeling techniques. However, only one set of GA parameters was used for the optimization, making it the main limitation of this research study. For future studies, it is suggested to apply other combinations of the GA parameters and compare their performance to find the most optimum setting. With other metaheuristic algorithms, such as PSO, GA could be used on a more extensive dataset with the ICD-diagnosis code added to the input variables. Previous studies that have used diagnostic ICD codes in their research study have models with a prediction accuracy of over 80% [10, 16, 17]. Improving the fitness function of XGBoost by simultaneously including dispersion indices and the mean of errors is another idea to work on and improve the results for practical uses. GA could also be used to optimize deep learning models such as ANN, which in future studies can be investigated more deeply.

## Figures and Tables

**Figure 1:** One-hot coding of four categorical features.

**Figure 2:** Boxplot diagram of absolute errors of predictive models.

**Figure 3:** Predicted values (*Y*-axis) vs. actual values (*X*-axis) of LOS for models: (a) KNN. (b) Lm. (c) Lm_transformed. (d) DT_default. (e) DT_GA. (f) ANN. (g) XGB_default. (h) XGB_GA. (i) RF_default. (j) RF_GA.

**Figure 4:** Relative comparison of errors statistical indices.

**Table 1:** Details of reviewed studies.

Ref.	Sample	LOS type		Predictive method^*∗*^∗			HPO	Best model	Validation indicator	
		Continuous	Categorical	Regression	Machine learning	Deep learning				
[13]	All admitted patients	*∗*	—	MR	—	—	—	MR	*R * ^2^	0.267
[14]	ICU-following cardiac surgery patients	—	*∗*	LR	—	—	—	LR	Accuracy	0.79
[10]	Diabetic patients	—	*∗*	GLM-NB	RF-GBM	ANN	Various experiments	Ensemble	AUC	0.81
[17]	Newborns	—	*∗*	NB- LR- MLP	DT-RF-R and.T-SVM	—	Not mentioned	RF	AUC	0.87
[4]	Cardiac patients	—	*∗*	—	RF-SVM-BN	ANN	Not mentioned	RF	Accuracy	0.8
[12]	Neurosurgery patients	*∗*	—	—	—	RNN-GRU	—	RNN-GRU	MAE	2.8
[15]	Radical cystectomy for muscle-invasive bladder cancer	*∗*	—	GLM	—	—	—	GLM	*R * ^2^	0.048
[11]	Brain tumor surgery patients	—	*∗*	Regression-based models	Tree-based models	ANN	Grid search	Ensemble	RMSE	0.5
[16]	Elective patients	—	*∗*	NB-BN -KNN- Kstar- LWL	C4.5 DT-SVM-decision table		Not mentioned	BN	AUC	0.9
[18]	ICU	—	*∗*	FL -KNN-Rerg.T-NB	CT-TB-RF-SVM	ANN	Not mentioned	FL	Accuracy	0.92
[20]	COVID-19 patients	*∗*	—	—	DT	—	Not mentioned	DT	MAE	2.84
[21]	Inpatients	—	*∗*	NB- KNN	DT -SVM,-XGBoost- nonlinear weighted XGBoost	—	Grid search	Nonlinear weighted XGBoost	RMSE	1.52
[13]	Lung cancer patients	—	*∗*	LR	RF- XGBoost	—	Not performed	RF	—	—

^*∗*^Methods. BL, binary logistic; BN, Bayesian network; FL, fuzzy logic; GLM, generalized linear model; KNN, K-nearest neighbors; LR, logistic regression; LWL, locally weighted learning; MLP, multilayer perceptron; MR, multiple regression; NB, Naïve Bayes; Reg.T, regression tree; CT, classification trees; DT, decision tree (J48); GBM, gradient boosting machine; Rand.T, random tree; RF, random forest; SVM, support vector machines; TB, tree bagger; ANN, artificial neural network; GRU, gated recurrent unit; RNN, recurrent neuronal network.

**Table 2:** Potential variables affecting LOS.

No.	Author	Ref.	Age	Sex	Insurance	Marital status	Medical advice number	Physician's expertise level
1	Baek et al., 2018	[13]			*∗*		*∗*	
2	Meadows et al., 2018	[14]	*∗*	*∗*				
3	Alahmar et al., 2018	[10]	*∗*	*∗*				
4	Thompson et al., 2018	[17]		*∗*	*∗*			
5	Daghistani et al., 2019	[4]	*∗*	*∗*				*∗*
6	Danilov et al., 2019	[12]						
7	Ray-Zack et al., 2019	[15]	*∗*	*∗*		*∗*		
8	Muhlestein et al., 2019	[11]	*∗*	*∗*				
9	Steele and Thompson, 2019	[16]	*∗*	*∗*	*∗*			
10	Abd-Elrazek et al., 2019	[18]	*∗*	*∗*				
11	Mahboub et al., 2021	[20]	*∗*	*∗*				
12	Alsinglawi et al., 2022	[21]	*∗*					

**Table 3:** Statistical characteristics of variables in the studied sample.

No.	Variable	*n*	Mean ± SD/percent
1	Age (year)	200	63 ± 19
2	Sex		
3	Female	100	50%
4	Male	100	50%
5	Marital status		
6	Married	179	90%
7	Single	21	11%
8	Main insurance type		
9	Ordinary social security insurance (ordinary SSI)	180	90%
10	Occupational social security insurance (occupational SSI)	5	3%
11	Employee health insurance (employee HI)	3	2%
12	Special social security insurance (special SSI)	6	3%
13	Without insurance (without insurance)	6	3%
14	Physician expertise level		
15	General practitioner	90	45%
16	Specialist	107	54%
17	Subspecialty physician	3	2%
18	Medical advice no		2 ± 3
19	LOS (day)		5.6 ± 3.4

**Table 4:** Correlation between independent variables and LOS.

No.	Variable	Correlation	*p* value	*p* value < 0.05
1	Age	−0.06	0.4032	
2	Medical advice number	0.46	0.0001	<0.05
3	Sex_F	0.02	0.7823	
4	Marital status_married	−0.04	0.5808	
5	Main insurance type_employee HI	0.20	0.0066	<0.05
6	Main insurance type_occupational SSI	0.08	0.2579	
7	Main insurance type_ordinary SSI	0.02	0.7514	
8	Main insurance type_special SSI	−0.05	0.4677	
9	Main insurance type_without insurance	−0.16	0.0291	<0.05
10	Physician expertise level_general practitioner	0.02	0.7447	
11	Physician expertise level_specialist	−0.07	0.3696	
12	Physician expertise level_subspecialty physician	0.17	0.0206	<0.05

**Table 5:** Hyperparameters of tree-based models in the training model and genetic algorithm.

Model	Hyperparameters	Type	Interval	Training model	Genetic algorithm	
				Default	Interval	Optimized
Decision tree	max_depth	Int	—	None	(1, 1000)	224
	min_samples_leaf	Int	—	1	(1, 50)	17
	ccp_alpha	Nonnegative float	—	0	(0, 1)	0.9

Random forest	max_features	Int	(1, no. of variables)	1	(1, 12)	6
	n_estimators	Int	(1, inf)	1	(50, 1000)	883
	max_depth	Int	(1, 100)	100	(1, 7)	43
	min_samples_leaf	Int	(1, sample size)	—	(1, 50)	8
	max_samples	Float	(0,1)	1	(0.1, 1)	0.65

XGBoost	learning_rate	Float	(0,1)	0.3	(0.001, 1)	0.4
	n_estimator	Int	(1-Inf)	1000	(50, 1000)	139
	max_depth	Int	(0, inf)	6	(1, 7)	1
	Subsample	Float	(0-1)	1	(0.1, 1)	0.9
	colsample_by_tree	Float	(0-1)	1	(0.1, 1)	0.15
	reg_lambda	Nonnegative float	—	1	(1, 3)	2.8

**Table 6:** Mechanism of tree-based HPO with GA.

**Input:** Number of folds for cross-validation*K*, dataset *D*, number of generations *G*, population size *P*, crossover probability CP, and mutation probability MP
**Output:** the optimum value of tree-based models hyperparameter
*g* = 0
Initialize population randomly of size *P*
**While ** *g* < *G* do:
*g* = *g* + 1
**For ***p* = 1 to *P* do:
Use the GA solutions for tree-based hyperparameters from the *p*th individual
**For ***k* = 1 to *K* do:
Divide *D* into *K* parts, 1 part as the testing set Test-*S* and (*K* − 1) parts as the
training set Train-*S*
Train the tree-based model on the training set Train-S
Predict the test set Test-*S* using the trained tree-based model
Calculate the mean square errors (MSEs)
**End for**
Calculate the value of the fitness function based on calculated MSEs
**End for**
Select 2 individuals by the steady-state selection method
Use the uniform crossover operator with the probability CP on selected individuals
Use the mutation operator with the probability MP on a new individual
Add the new individual to the population
**End while**
Return the optimum hyperparameter values of tree-based models

**Table 7:** Absolute error indices of predictive models on the test dataset.

No.	Model	Mean (day)	Median (day)	SD (day)	IQR (day)	Min (day)	Max (day)
1	KNN	1.78	1.75	1.50	1.75	0.00	6.33
2	Lm	1.56	1.33	1.14	1.56	0.00	4.56
3	Lm_transformed	1.52	1.19	1.26	1.37	0.10	5.19
4	DT_default	2.15	2.00	1.79	1.00	0.00	7.00
5	DT_GA	1.95	1.65	1.61	2.00	0.35	6.35
6	RF_default	1.65	1.02	1.47	1.87	0.09	5.71
7	RF_GA	1.76	1.34	1.42	1.50	0.04	5.57
8	XGBoost_default	2.45	2.56	1.93	2.54	0.00	7.67
9	XGBoost_GA	1.54	1.14	1.38	1.26	0.04	5.68
10	ANN	1.61	1.20	1.20	1.75	0.03	4.71

**Table 8:** The percentage change of the absolute error in the GA-optimized models.

No.	Model	Mean (%)	Median (%)	SD (%)	IQR (%)	Min	Max (%)
1	DT_GA	−10	−17	−10	100	—	−9
2	RF_GA	7	31	−4	−20	—	−2
3	XGB_GA	−37	−56	−28	−50	—	−26

## Data Availability

The dataset used to support the findings of this study is available from the corresponding author upon request.
